# Involvement of the glutamate/glutamine cycle and glutamate transporter GLT-1 in antidepressant-like effects of Xiao Yao san on chronically stressed mice

This article has been retracted.

**DOI:** 10.1186/s12906-017-1830-0

**Published:** 2017-06-19

**Authors:** Xiu-Fang Ding, Yue-Hua Li, Jia-Xu Chen, Long-Ji Sun, Hai-Yan Jiao, Xin-Xin Wang, Yan Zhou

**Affiliations:** 1 School of Basic Medical Science, Beijing University of Chinese Medicine, Beijing, 100029 China; 2 Beijing Chaoyang Hospital, Capital Medical University, Beijing, 100043 China; 3 School of Basic Medicine, Henan University of TCM, Henan, 450046 Henan China

**Keywords:** Herbal medicine, Depression, Animal research

## Abstract

**Background:**

Xiao Yao San (XYS) is an herbal prescription which is used in the treatment of depression for thousands of years from Song dynasty in China (960–1127 A.D.), and is the bestselling and most popular herb formula for treating major depression. This study aimed to assess the chronic antidepressant effects of XYS and fluoxetine in depressed mice induced by chronic unpredictable mild stress (CUMS) and its association with  alterations in glutamate/glutamine cycle and glutamate transporters.

**Methods:**

Mice in the control and model group were given 0.5 ml physiological saline by intragastric administration. Mice in two treatment groups were given XYS (0.25 g/kg/d) and fluoxetine (2.6 mg/kg/d), respectively. The depressive-like behaviors such as forced swim test (FST), sucrose preference test (SPT) and novelty-suppressed feeding (NSF) test were measured after mice exposed to CUMS for 21 days. Body weight, contents of glutamate and glutamine, glutamine/glutamate ratio that is usually thought to reflect glutamate/glutamine cycle, and the protein and mRNA expressions of glutamate transporters (excitatory amino acid transporter 1–2,GLAST/EAAT1 and GLT-1/EAAT2) were measured. The immunoreactivities of GLAST and GLT-1 in the hippocampus were also investigated.

**Results:**

After CUMS exposure, mice exhibited depressive-like behaviors, body weight loss, increased glutamate level, decreased glutamine level, elevated glutamine/glutamate ratio, decreased GLT-1 protein expression and mRNA level, and decreased average optical density (AOD) of GLT-1 in the CA1, CA3 and DG in the hippocampus. These abnormalities could be effectively reversed by XYS or fluoxetine treatment. In addition, the study also found that GLAST expression in the hippocampus could not be altered by 21-d CUMS.

**Conclusion:**

The studies indicated that XYS may have therapeutic actions on depression-like behaviors induced by CUMS in mice possibly mediated by modulation of glutamate/glutamine cycle and glutamate transporter GLT-1 in the hippocampus.

## Background

Depression, a commonly occurring psychiatric condition, is a leading cause of disability and premature death worldwide. Furthermore, it is also closely related to economic healthcare costs [1]. As defined in the fifth edition of the Diagnostic and Statistical Manual (DSM-5), major depressive disorder (MDD) is associated with a loss of pleasure and the presence of depressed mood during social activities which are met by four criteria including changes in sleep, energy, concentration and appetite over a period of two weeks [2–4]. MDD is a highly prevalent chronic illness and psychiatric disorder affecting a rising percentage of the world’s population. More than 16% of adults experience MDD at some point during their lifetimes [5]. Consequently, the development of efficacious treatments for MDD is urgently needed [6].

Recently, in an effort to find treatments that can effectively improve the depressive state without unpleasant side effects commonly experienced with the use of western medicine treatments of MDD, much attention has been given to natural remedies, including traditional Chinese medicine (TCM) [7, 8]. Based on TCM theories and supported by clinical observations, patients with MDD commonly exhibit liver stagnation and spleen deficiency. XYS, an herbal prescription used since tenth century, has been used to treat MDD because of its ability to sooth the liver and tonify the spleen. Indeed, Butler and Pilkington showed that XYS was more effective than placebo [9]. Furthermore, XYS is the bestselling and most popular herbal formula used for treating major depression [7]. Clinical research demonstrates that XYS can significantly decrease the Hamilton depression scores of patients with MDD. Additionally, XYS was reported to improve depressive-like behaviors in rats through regulation of the mammalian target of rapamycin (mTOR) [10]. Moreover, we have previously shown that XYS treatment can effectively improve depressive-like behaviors in rats exposed to chronic immobilization stress (CIS) through the inhibition of LC-NE neuronal activity [11]. Although the therapeutic mechanism of XYS on depression has been explored and shown to be related to the nervous system, to our knowledge, few studies have demonstrated an association between the antidepressant-like effects of XYS and glutamatergic system in depressed rodents.

The evidence shows the involvement of the glutamatergic system in the biological mechanisms of MDD. In glutamate metabolism, unlike the monoamine transmitter that is transported into presynaptic nerve terminals, Glutamate (Glu) is predominately cleared by glial cells through the excitatory amino acid transporters (EAATs). While monoamine metabolism leads to excreted waste products, Glu is recycled efficiently through the glutamate/glutamine (Glu/Gln) cycle. Glu is quickly converted into the ‘inert’ intermediate, glutamine (Gln), within glial cells by the enzyme glutamine synthetase (GS) after uptake by EAATs. Subsequently, Gln is transferred to neurons where it is converted back into Glu, and packaged into synaptic vesicles by several vesicular glutamate transporters [12]. Glu and Gln are key participants in the Glu/Gln cycle and are highly involved in the pathophysiological processes underlying mood disorders. Glutamate levels in the central nervous system (CNS) are mainly regulated through a family of EAATs localized on astroglia and neurons. EAATs play a critical role in the Glu/Gln cycle, as they maintain low basal levels of glutamate in the synapse, and facilitate receptor-mediated responses to glutamate release [13, 14]. To date, five distinct sodium-dependent, high-affinity glutamate transporters from human and animal tissues, have been cloned [EAAT1 (GLAST in rodent), EAAT2 (GLT-1 in rodent), EAAT3 (EAAC1), EAAT4 and EAAT5)]. These types of EAAT transporters differ in tissue distribution, molecular structure and pharmacological properties [15, 16]. Interestingly, reduced levels of astrocyte-specific EAATs (EAAT1 and EAAT2) were detected in the brains of depressed patients [17] and animal models [18]. Thus, measurement of these amino acids and glutamate transporters in depressed rodents can potentially aid our understanding of the role that the glutamatergic system plays in depression.

In the present study, using the CUMS model (define CUMS) we investigated whether alterations in the glutamatergic system occur specifically within the hippocampus and have a part in the pathology of MDD as well as explain therapeutic responses to the antidepressant actions of XYS. Specifically, behavioral tests (FST, SPT and NSF define test) and body weight with CUMS were evaluated in mice. The amounts of Glu and Gln in the hippocampus were measured, and the Gln/Glu ratios were calculated, as these ratios are considered to reflect the degree of Glu/Gln cycle involvement in neuron-glia communication in the synapses. In addition, protein and mRNA expression, along with the immunoreactivities of glutamate transporters, GLAST and GLT-1, were measured.

## Methods

### Preparation of XYS

The XYS formula was composed of eight herbal medicines. The composition and dose of the prescription is listed in Table 1. The raw herbs were obtained from the Tongrentang (Bozhou, Anhui, China) Decoction Pieces Limited Company, and then authenticated by Dr. B. Liu (department of Botany of Beijing, University of Chinese Medicine). The drugs were extracted by the Chinese medicine preparation room of China-Japan Friendship Hospital as previously described [19]. The extraction rate was 18.8%, and the quality control of XYS was identified by high-performance liquid chromatography-mass spectrometry analysis (LC-MS/MS).

**Table 1:** Composition of XYS

Medicinal plant	Amount (g)
Poria((Poria cocos (Schw.) Wolf))	15
Rhizoma Zingiberis Recens (*Zingiber officinale* Rosc.)	15
Radix Angelicae Sinensis (Angelica sinensis (Oliv.) Diels)	15
Rhizoma Atractylodis Macrocephalae (Atractylodes macrocephala Koidz.)	15
Radix Paeoniae Alba (*Paeonia lactiflora* Pall.)	15
Radix Glycyrrhizae (Glycyrrhiza uralensis Fisch.),	6
Herba Menthae (Mentha haplocalyx Briq.)	6
Radix Bupleuri (Bupleurum chinense DC.)	15

### LC-MS/MS measurement for XYS

The eight compounds, including Palmitic acid, AtractylenolideII, Curcumin, Paeoniflorin, Ligustilide, Saikosaponin D+ B1 and Pachymic acid in XYS were examined. The molecular structures of these ingredients are shown in Fig. 1. Standards of Palmitic acid (purity ≥ 99.2%), Curcumin (purity ≥ 98.12%), Paeoniflorin (purity ≥ 98.78%), Liquiritin (purity ≥ 98.68%), Atractylenolide II (purity ≥ 99.50%), Saikosaponin B1 (purity ≥ 99.53%), Saikosaponin D (purity ≥ 98.55%) and Pachymic acid (purity ≥ 98.83%) were obtained from the Chengmust Company (Sichuan Province, China). LC-MS/MS analysis was performed by using a 5500 QTRAP LC-MS/MS system (AB SCIEX, Framingham, MA, USA). In the positive ionization mode, the MS parameters of curtain gas (CUR), collisionally activated dissociation gas (CAD), collision cell entrance potential (CXP), declustering potential (DP), nebulizer gas (GS1), entrance potential (EP) and GS2 (heater gas) were set to 40, medium, 13, 120, 50, 10 and 50, respectively. The mobile phase A consisted of 0.1% formic acid and water, and mobile phase B consisted of methanol. The gradient program is shown in Table 2. In the negative ionization mode, the MS parameters of CUR, CAD, CXP, DP, GSI, EP and GS2 were set to 40, medium,-16, −90, 50, −10 and 50, respectively. The mobile phase A consisted of 0.1% formic acid and water, and mobile phase B consisted of methanol. The gradient program is shown in Table 2.

**Fig. 1:** Molecular structures of eight ingredients in XYS sample. **a** Palmitic acid. **b** Curcumin. **c** Paeoniflorin. **d** Liquiritin. **e** Atractylenolide II. **f** Saikosaponin D. **g** Saikosaponin B1. **h** Pachymic acid

**Table 2:** The gradient program in the positive and negative ionization mode

Lonization mode	Time(min)	Flow rate	A(%)	B(%)
Positive Ionization mode	0	300	90	10
	2	300	30	70
	3	300	20	80
	6.5	300	0	100
	6.6	300	90	10
	8.5	300	90	10
Negative ionization mode	0	300	90	10
	1	300	60	40
	2.2	300	40	60
	4	300	5	95
	5.5	300	5	95
	5.6	300	90	10
	8	300	90	10

### Validation of LC-MS/MS method

The method was measured for linearity, accuracy, precision, and stability according to the previous reports [20, 21].

### Linearity

The stock solutions were prepared by dissolving 5 mg of references into 5 mL methanol to a final concentration of 1 mg/mL. 100 μL of this solution was added methanol to a final concentration of 10 μg/mL. The working standard solutions were prepared via dilutions of the stock solution with methanol to obtain the following concentrations: 0.5, 1, 5, 10, 25, 50, and 100 ng/mL. These solutions were kept at 4 °C. Linearity of the method was evaluated by standard curves of eight ingredients ranging from 0.5 ng/ml to 100 ng/ml.

### Precision and accuracy

The precision and accuracy assays were carried out in six replicates at three quality control levels (low: 2 ng/mL; medium: 20 ng/mL;and high: 50 ng/mL) on the same day and on three consecutive days. The intra- and inter-day accuracy and precision of Palmitic acid, Curcumin, Paeoniflorin, Liquiritin, Atractylenolide II, Saikosaponin D**,** Saikosaponin B1 and Pachymic acid were examined to represent the intra- and inter-day accuracy and precision of XYS samples. The relative standard deviation (RSD%) values of six XYS samples were used to report the precision. The accuracy was measured via comparing the calculated concentrations from the standard curves with the theoretical concentrations.

### Stability studies

The stability of XYS was conducted on triplicate at three quality control levels (low: 2 ng/mL;medium: 20 ng/mL; and high: 50 ng/mL). The first set was assayed immediately and used as a reference point after reinjection of the same sample at 0,2,4,8,12, and 24 h, and the solutions were kept at room temperature in the auto-sampler tray. The stability was assessed from RSD% according to the peak area of eight ingredients in XYS samples.

### The contents determination of XYS

The contents of eight ingredients in XYS were calculated by using the external standard method. Approximately 0.2 g of the XYS was dissolved in 1 ml of methanol, and the mixture was vortexed. After centrifuging at 12, 000 x g for 5 min, 50 μL of the sample supernatant was added 950 μL of methanol, and the mixture was vortexed well before injection into the LC-MS/MS system for analysis.

### Animals

The specific pathogen-free (SPF) mice (aged: 12 weeks, NO.SCXK 2012–0001) were obtained from Beijing vital River of Charles River company, the distributor of the Jackson Laboratory (USA). All animals were housed within standard animal rooms (room temperature: 21 ± 1 °C; light condition: a 12 h/12 h dark/light cycle; relative humidity: 30%–40%). The mice were allowed to acclimatize for at least 1 week before the experiments commenced. A total of 60 mice were arbitrarily assigned into four groups based upon their weight, namely, control group (no-stress +physiological saline), model group (21-d CUMS +physiological saline), XYS treatment group (21-d CUMS + XYS), and fluoxetine (FLU) treatment group (21-d CUMS + FLU). All mice were housed singly in cages, and the protocol in this experiment adhered strictly to the guidelines for the Care and Use of Laboratory Animals of China, and was approved by the Animal Ethics Committee of Beijing University of Chinese Medicine. All efforts were aimed to minimize animal suffering.

### Drugs

Mice in the control and model group were given 0.5 ml physiological saline by intragastric administration. Mice in the two treatment groups were given XYS (0.25 g/kg/d) and FLU (2.6 mg/kg/d), respectively. The medium dose of XYS (0.25 g/kg/d) was selected for its small dosage with satisfactory efficacy based on previously reported findings [20, 22]. The physiological saline or drugs were intragastrically administered for 21 days.

### CUMS paradigm

All animals were subjected to CUMS for 21 days except the control group mice. The CUMS paradigm was performed as previously reported [23] and some improvements were made. This protocol involves a variety of mild stressors: (1) restraint stress for 3 h, (2) empty cage for 24 h, (3) wet and soiled cage for 24 h, (4) cold swimming at 10 °C for 5 min, (5) food deprivation for 24 h, (6) water deprivation for 24 h, (7) crowded cage for 24 h. These stimulations were randomly arranged for one type of stimulation per day with no repeat of the same stimulation on continuous days, which guaranteed animals would receive unpredictable stimulations. Body weight was recorded on day 0 (before the onset of experiments), day 7, day 14 and day 21 during stress period. The body weight and SPT were recorded weekly, and other behavioral assessments (FST and NSF) were performed after the last stimulation.

### Sucrose preference test (SPT)

The SPT test was performed weekly during the stress period, and followed a reported procedure with minor modifications [11, 24]. Briefly, mice were had 24 h access to a palatable 1% sucrose solution (Biotech, #0335), followed by 24 h of water deprivation and a 4 h exposure to two identical bottles, one filled with 1% sucrose solution and the other with water. Sucrose preference was defined as the ratio of the volume of sucrose versus water consumed during the 4-h test.

### Forced swimming test (FST)

As previously described [24, 25], mice were individually placed into a clear glass cylinder (height; 24 cm, diameter; 19 cm), which was filled to 20 cm of water at room temperature (23 ± 1 °C). Immobility time was measured for 6 min using a video. The duration of immobility for each mouse was recorded during the final 5 min by experimenters who were blinded to the experimental design.

### Novelty suppressed feeding (NSF) test

The NSF test was performed at day 21. Mice were deprived from food for 24 h prior to the test, while water was provided ad libitum. A small piece of mouse chow was placed in the center of the arena in a Plexiglas box (25 cm × 25 cm × 20 cm). Mice were placed in the corner of the testing arena, and the time of the first feeding episode was recorded [26]. Once the mouse began to bite the chow, the tested animal was immediately removed to a single house cage. The amount of food consumed in the subsequent five minutes was measured.

### Tissue sample collection

The mice were sacrificed by decapitation after behavioral tests. The bilateral hippocampus of five mice in each group were removed immediately on ice, and placed in liquid nitrogen for rapidly freezing and stored at −80 °C for LC-MS/MS measurement. The other five mice in each group were decapitated; the left hippocampi were removed immediately on ice, and also placed in liquid nitrogen for rapidly freezing and then stored at −80 °C for protein analysis. The right hippocampi of the remaining mice were kept in 10 volumes of RNA later Solution (Biotech, #2714 k) for quantitative real-time fluorescence polymerase chain reaction (qRT-PCR) assay. The whole brains of the remaining mice in each group were removed after accepting heart perfusion. The brains were fixed in 4% paraformaldehyde (PFA) solution (4% PFA, 2.5% glutaraldehyde, and 0.1 mol PBS) for immunohistochemistry.

### LC-MS/MS analysis

The hippocampal samples were prepared as previously reported [27], with minor modifications. Hippocampus was homogenized by adding 10-fold volume of 50% methanol (methanol: water = 1:1 *v*/v) and vortexed for 30s.The homogenates were then centrifuged at 12,000 g for 5 min at 4 °C. 5 μL of the supernatant was collected, and injected into the LC-MS/MS system for analysis.

The levels of Gln and Glu in the hippocampus were measured by an external standard method. The reference standards, including Gln and Glu were purchased from Sigma-Aldrich (2500 μM). The working standard solutions were prepared via dilution of stock solution with double distilled H_2_O to obtain the following concentrations: 0.25, 1.25, 2.25, 5 and 12.5 μM. These solutions were stored at 4 °C. The BEH T3 column (2.1 mm × 100 mm, 1.7 μm) was used for chromatographic separations. The temperature of the column was kept at 45 °C.The following gradient program was used to analyze the mobile phase consisting of solvent A (0.01% TFA in water) and solvent B (0.01% TFA in methanol): 0–1 min: 100% A;1–4 min: 100% A; 4–6 min: 90% A,10% B; 6–10 min: 80% A, 20% B; 10–12 min: 50% A, 50% B; 12–14 min: 100% B. The flow rate was 0.25 mL/min and the injection volume was 5 μL.

### Western blotting analysis

Protein levels of GLAST and GLT-1 were measured by Western blotting analysis. The procedure was performed as previously described [11, 25]. Briefly, proteins were extracted from hippocampal tissue, and protein concentrations were measured using a BCA protein assay kit (Beyotime, Shanghai, China). The lysates were loaded onto 12% SDS-PAGE gels for separation, electro-transferred onto PVDF (polyvinylidene fluoride) membranes, and blocked in PBST with 5% nonfat milk. The membranes were incubated with primary antibodies at 4 °C overnight [(GLAST, Cell signaling, #5684, 1:1000; GLT-1, Abcam, #69098, 1:1000), and anti-β-actin (Santa Cruz Biotech, 1:2000)]. After washing with PBST three times for 5 min each time, membranes were incubated with horseradish peroxidase-(HRP-) conjugated secondary antibody. Membranes were developed using the enhanced chemi-luminescence (ECL) detection reagent for 3 min. The optical density of protein band was measured using the Image J software.

### qRT-PCR analysis

Total RNA was extracted using Trizol® reagent (Invitrogen). The RNA from each sample was used to synthesize cDNA using High Capacity cDNA Reverse Transcription Kit with Gene Amp PCR System (Applied Biosystems, USA). The sequences for primers were as follows: GAPDH,5′-GGCAAATTCAACGGCACAGT-3′;3′-ACGACATACTCAGCACCGGC-5′;GLAST,5′-AATGTGGTATGCGCCTCTGG-3′;3′-GCAGCAACCCTCCAATGAAA-5′;GLT-1,GTGGCACCTCCATCTGAGGA,3′-CACCATCAGCTTGGCCTGTT-5′.qRT-PCR was performed on an ABI ViiA7 Real-Time PCR System (Applied Biosystems,USA) and an SYBR® Green PCR Master Mix in a final volume of 20 μl with the following thermal cycling conditions: 95 °C for 1 min, followed by 40 cycles of 95 °C for 2 min, 94 °C for 10 s,59 °C for 10 s, and 72 °C for 40 s. mRNA expressions were quantified by subtracting the threshold cycle GAPDH(C_t_) value from the C_t_ value of the genes of interest. It was expressed as 2^-△△^C_t_.

### Immunohistochemical staining

Immunohistochemistry staining was carried out according to the method previously described [11]. The brains were fixed in 4% PFA solution for 48 h and were then cut into serial sections (5 μm). The paraffin-embedded hippocampal sections were processed as free-floating slices, including deparaffinized, rehydrated, and pretreated with hydrogen peroxidase. Antigen retrieval was performed by heating in 0.01 mmol/L citrate buffer (PH = 7.2) for 15 min. Slices were incubated with primary antibodies (GLAST, Cell signaling, #5684, 1:50; GLT-1, Abcam, #69098, 1:300) after blocking in the antisera. After incubation with the secondary antibody, sections were placed in DAB reagent (#00–2014, Invitrogen, USA) for 5–10 min at room temperature. After a further rinsing in 0.1 mol PBS, sections were restained with hematoxylin, and were mounted on gelatine-coated slides for observation. The images of the positively stained expressions in the CA1, CA3 and DG regions of the hippocampus were captured at 200 x magnifications by an Olympus BX 41 microscope.

### Statistical analysis

All data were expressed as mean ± standard error of the mean (S.E.M) and analyzed using SPSS 17.0 software. The mean values were conducted using one-way analysis of variance (ANOVA) followed by the least significant difference(LSD) test for post hoc comparisons when equal variances were assumed. Analyses of variance with repeated measures were used to compare the body weight. Values of F, degrees of freedom and levels of significance were reported in the results section. Values of *P* < 0.05 were considered statistically significant.

## Results

### Quality control of XYS by LC-MS/MS

In order to investigate the quality control of XYS, the samples were identified by high-performance liquid chromatography-mass spectrometry analysis (LC-MS/MS). The method was validated according to the US Food and Drug Administration bioanalytical method validation(BMV) guidance, including linearity, precision, accuracy, and stability [21].

The standard curves were linear over the concentration ranges of 0.5–100 ng/ml for ingredients. The results of Table 3 show a good linearity according to Pharmacopoeia guidelines. The mean concentrations of Palmitic acid, Curcumin, Paeoniflorin, Liquiritin, Atractylenolide II, Saikosaponin +Saikosaponin B1 and Pachymic acid in XYS samples were 1062, 0.084, 5462.000, 828.500, 16.160, and 112.60,3.114 ng/ml, respectively (Table 3). The alignment of ingredients in XYS samples could match the corresponding peaks of XYS by the same LC-MS/MS elution system (Fig. 2), indicating these ingredients might be quality control references of XYS.

**Table 3:** Linearity and concentrations of eight ingredients in XYS sample

Analytes	Regression equation	Correlation Coefficient(r)	Concentration (ng/ml)
Palmitic acid	y = 16,615.90166× + 7951.53113	0.99945	1062.000
Curcumin	y = 5.38124e4x-745. 66,733	0.99455	0.084
Paeoniflorin	y = 1265.39220× + 2690.13765	0.99765	5462.000
Liquiritin	y = 5.16820e4x + 1679.84738	0.99681	828.500
Atractylenolide II	y = 1.69650.e5x + 19,343.32087	0.99309	16.160
SaikosaponinD+ B1	y = 7746.04828×-408.30435	0.99549	112.60
Pachymic acid	y = 6398.24497× + 1712.95158	0.99802	3.114

**Fig. 2:** The chromatograms of eight ingredients in XYS sample. **a** Palmitic acid. **b** Curcumin. **c** Paeoniflorin. **d** Liquiritin. **e** Atractylenolide II. **f** Saikosaponin D + SaikosaponinB1. **g** Pachymic acid. References results are shown on the left side, and results on samples are shown on the right side

The inter- and intra-day precision and accuracy in six XYS samples were examined. Precision was based on the calculation of RSD%(Relative Standard Derivation, RSD). The intra-day precision ranged from 1% to 4.02%, and the inter-day precision ranged from 2.22% to 3.47% (Table 4). The intra-day accuracy ranged from 90.2% to 108.5%, and the inter-day accuracy ranged from 95.3% to 108.9%(Table 4). The inter- and intra-day precision and accuracy data of the assays were within the acceptable criteria, indicating that the reliability of method developed.

**Table 4:** Precision, accuracy and stability in XYS sample

Analytes	Precision (RSD%)		Accuracy (%)		Stability (RSD%)
	Intra-day	Inter-day	Intra-day	Inter-day	
Palmitic acid	3.59	2.61	100.1–109.2	98.5–100.4	3.31
Curcumin	3.69	2.19	103.2–107.4	101.7–107.1	8.64
Paeoniflorin	2.88	2.88	97.8.3–104.1	96.6–101.8	4.81
Liquiritin	4.02	3.47	98.2–108.5	99.4–106.3	1.90
Atractylenolide II	2.86	2.73	99.8.3–107.1	98.6–101.2	1.75
Saikosaponin D+ B1	1.06	2.95	94.2–110.5	9742–108.9	6.76
Pachymic acid	1.06	2.69	95.2–107.5	96.5.-107.4	4.53

Stability was assessed from RSD% according to the peak area of ingredients in XYS at 0, 2, 4, 8, 12, and 24 h. The RSD% values of Palmitic acid, Curcumin, Paeoniflorin, Liquiritin, Atractylenolide II, Saikosaponin +Saikosaponin B1 and Pachymic acid were 3.31%, 8.64%, 4.81%, 1.9%, 1.75%, 6.76% and 4.53%, respectively (Table 4). The results showed that the analytes were stable at room temperature for 24 h with RSD all less than 15%.

### XYS improved body weight in mice exposed to CUMS

In order to observe the variation of body weight in mice subjected to CUMS, body weight in each mouse was measured before the onset of the CUMS regimen and then weekly until the end of CUMS procedure. CUMS mice showed a reduction in body weight at the third week (Fig. 3a, f (3, 56) =5.568, *P* < 0.001). While XYS or FLU treatment significantly increased the body weight compared with the model group (both *P* < 0.05).

**Fig. 3:** Effects of XYS on body weight and behaviors in mice with CUMS. **a** Body weight was recorded once a week during 21d–CIS period. **b** The forced swimming test(FST) was conduct on day 21. **c**, **d** Sucrose preference test(SPT) was performed weekly. **e**, **f** The Novelty suppressed feeding (NSF) test was performed on day 21. Data were expressed as mean ± S.E.M, *n* = 15 per group. ^∗^ *P* < 0.05, ^∗∗^ *p* < 0.001 vs. control; ^△^ *p* < 0.05, ^△△^ *p* < 0.001 vs. model

### XYS alleviated depressive-like behaviors in mice exposed to CUMS

In order to evaluate depressive-like behaviors in mice exposed to CUMS, several behavioral tests were carried out, including FST, SPT and NSF test. The forced swimming test which evaluated the efficacy of antidepressant drugs showed that the immobility time in the model group mice was significantly longer than those of control group mice after modeling for 21 days (Fig. 3b, f (3, 56) =3.959, *P* < 0.05). In contrast, the immobility time was significantly shortened after XYS treatment as compared with the model group (*P* < 0.05), and similar result was also observed in mice treated with FLU (*P* < 0.001). Additionally, these two treatments effects were also accompanied by increased swimming behavior. Anhedonia, which is defined by the reduced preference for sucrose, is the key symptom of depression, and is used for observing the depressive-like states in rodents [28]. To examine the dynamics of the CUMS response, the sucrose preference of each mouse was recorded weekly. Initially, all mice had a similar sucrose preference in a baseline condition on day 0 (before stress, Fig. 3c, f (3, 56) =0.934, *P* > 0.05). On the other hand, a significant drop of sucrose preference was measured after 3 weeks of stress (Fig. 3d, f (3, 56) =48.983, *P* < 0.001). In contrast, XYS or FLU treatment reversed this reduction and significantly increased the sucrose preference when compared with the model group (both *P* < 0.001). In the NSF test, CUMS mice had longer latencies to bite the chow than the control animals, and had a significant difference (Fig. 3e, f (3, 56) =4.065, *P* < 0.05). Compared to the model group, this increased latency was significantly attenuated by XYS or FLU administration (both *P* < 0.05)*.* The CUMS exposed mice also significantly consumed less food (Fig. 3f, f (3, 56) =34.102, *P* < 0.001). These changes reversed by XYS or FLU treatment (both *P* < 0.001).

### XYS reversed the effects of CUMS on Glu/Gln cycle

To investigate whether XYS administration altered the Glu/Gln cycle in animal model of depression, the contents of Glu and Gln in the hippocampus were determined by LC-MS/MS. In this experiment, standard curves were constructed by plotting the peak area of the gradient concentrations of the two reference standards. The standard curves were linear over the concentration ranges of 0.25–12.5 μM for Glu and Gln. The calibration curves were as follows: y = 1.00896e6x + 16,712.02651 (R^2^ = 0.99967, Glu) and y = 3.60002e5 x + 16,942.46716 (R^2^ = 0.99987, Gln). The chromatograms of Glu and Gln are shown in Fig. 4a-b. An increased level of Glu was observed in the model group when compared with the control group (Fig. 4c, f (3, 16) =14.523, *P* < 0.05). This alternation could be effectively restored by the administration of XYS or FLU (both *P* < 0.05). In contrast, the levels of Gln in the model group was decreased compared with the controls, and there was a significant difference (Fig. 4c, f (3, 16) =10.780, *P* < 0.05). After administration of antidepressants, this reduction could be effectively restored with XYS and FLU treatment (*P* < 0.05, *P* < 0.01, respectively). An elevated Gln/Glu ratio was observed in stressed mice (Fig. 4d, f (3, 16) =13.173, *P* < 0.001), and was down-regulated by both XYS and FLU treatment (both *P* < 0.001).

**Fig. 4:** Alterations of contents of Glu and Gln, and the Gln/Glu ratio in the hippocampi of mice by CUMS as well as XYS and FLU treatment. **a** Chromatograms of Glu. **b** Chromatograms of Gln. Results on references are shown on the left side, and results on hippocampal samples are shown on the right side. **c** The contents of Glu and Gln in the hippocampi were detected by LC-MS/MS. **d** The glutamate/glutamine ratio was calculated. Data were expressed as mean ± S.E.M,*n* = 5 per group.^∗^ *P* < 0.05,^△△^ *P* < 0.01,^#^ *P* < 0.001 vs. control; ^△^ *P* < 0.05, ^##^ *P* < 0.001 vs. model

### XYS improved glutamate transporter expression in the hippocampi of CUMS mice

To investigate whether XYS altered the levels of glutamate transporters in an animal model of depression, the expressions of GLT-1 and GLAST were determined. First, we analyzed the effects of XYS on protein and mRNA levels of GLT-1 and GLAST in the hippocampi of CUMS mice. As shown in Fig. 5a, the CUMS exposure resulted in a significant decreases in protein levels of GLT-1 when compared with the control group (Fig. 5a, f (3, 16) =19.274, *P* < 0.01). In comparison with the model group, both XYS and FLU treatment significantly elevated GLT-1 protein expression (*P* < 0.05, *P* < 0.01, respectively). As shown in Fig. 5b, a similar tendency was observed for mRNA expression. The mRNA level of GLT-1 was significantly decreased in CUMS mice when compared with the control group (Fig. 5b, f (3,16) = 24.363, *P* < 0.01). These reductions were significantly restored to normal levels by XYS and FLU administration compared to CUMS mice (both *P* < 0.01). In addition, the effect of CUMS on protein and mRNA levels of GLAST was not changed (Fig. 5c, d). We further examined the effects of CUMS and XYS on the expression levels of GLAST and GLT-1 in the three hippocampal subregions using immunohistochemical staining. As shown in Fig. 6a, the average optical density (AOD) of GLAST in the CA1, CA3 and DG were not significantly reduced when compared with the control group. Compared with no-stressed mice, significant reductions of the AOD of GLT-1 in the three hippocampal subregions were measured and had significant differences (Fig. 6b, CA1:F(3,16) = 7.189, *P* < 0.05;CA3:F(3,16) = 10.907, *P* < 0.05; DG: F(3,16) = 11.219, *P* < 0.05, respectively). Increased AOD of GLT-1 in CA1, CA3 and DG were investigated after administration of XYS (*P* < 0.05, *P* < 0.05, *P* < 0.01, respectively). Similar results were also observed in mice treated with FLU (*P* < 0.05, *P* < 0.01, *P* < 0.01, respectively).

**Fig. 5:** Alterations of protein and mRNA expressions of GLAST and GLT-1 in the hippocampi of mice by CUMS as well as XYS and FLU treatment. **a**, **c** The protein expressions of GLT-1 and GLAST were measured by Western blotting. **b**, **d** The mRNAs levels of GLT-1 and GLAST were measured by qRT-PCR. Data were expressed as mean ± S.E.M, *n* = 5 per group.^∗∗^ *p* < 0.001 vs. control;^△^ *p* < 0.05,^#^ *p* < 0.01 vs. model

**Fig. 6:** Alterations of GLAST and GLT-1 immunoreactivities in the hippocampi of mice by CUMS as well as XYS and FLU treatment. **a**, **b** The AOD of GLAST and GLT-1 in the hippocampal subregions CA1,CA3 and DG were determined by immunohistochemical staining. Abbreviations:CA1 and CA3: hippocampal subregions of ammons horn (cornu ammonis), DG:dentate gyrus. Data were expressed as mean ± S.E.M,*n* = 5 per group.^∗^ *P* < 0.05 vs. control;^△^ *p* < 0.05, ^#^ *p* < 0.01 vs. model

## Discussion

Between 20%–50% of the population worldwide is afflicted with depression. Importantly, not all patients that experienced depression respond well to the current antidepressants, such as monoamine oxidase inhibitors, norepinephrine selective reuptake inhibitors. Furthermore, continuous treatment for at least several weeks or up to months is need for a full therapeutic response [29]. Some newer types of antidepressants are better tolerated and safer than older classes of antidepressants drugs, but they still frequently produce bothersome side-effects [30]. Therefore, seeking an effective intervention to treat depression is urgently needed. In the current study, an herbal formulation, XYS, was used and we focused on exploring the mechanism of its antidepressant effects on the glutamatergic system in the hippocampi of mice exposed to CUMS (used as an experimental model of depression).

In this study, to investigate the quality of XYS samples, the amounts of eight ingredients including Palmitic acid, Curcumin, Paeoniflorin, Liquiritin, Atractylenolide II, Saikosaponin D, Saikosaponin B1 and Pachymic acid were analyzed by LC-MS/MS. The results showed that the contents of the eight ingredients in the XYS samples were in concert with guidelines in Pharmacopoeia and had good quality control. Particularly, these samples were stable at room temperature for 24 h.

Rodents can timely adjust their physiological status under different kinds of stressful events. Excessive, chronic or long-term stress can result in body weight loss [19]. In the present study, body weight was not significantly different among groups after modeling for 7 days. CUMS started to affect body weight after modeling for 14 days and that affect led to a subsequent decrease by day 21. As expect, decreased body weight could be reversed by both XYS and FLU treatment. To assess the possible depressive behaviors in mice with CUMS, the FST, SPT and NSF tests were carried out. The forced swim test (FST, or called the Porsolt swim test), a rodent behavioral test, is used to evaluate the antidepressant efficacy of drugs, and experimental manipulation that is aimed at rendering depressive-like states [31]. Mice are placed in a glass tank that is filled with water and their immobility behaviors are recorded. Here, we found that the immobility time in mice exposed to CUMS for 21 days was significantly longer than controls; this was in contrast to the mice in XYS and FLU treatment group. In the SPT, anhedonia is conceptually thought as “a decreased capacity to experience pleasure of any sort” [32]. Here, a significant drop of sucrose preference was measured after 3-week stress, and was reversed by both XYS and FLU treatment. Particularly, this alteration tendency was consistent with the results in changes in body weight. Furthermore, we measured another type of depressive-like behavior, the appetite in NSF test, which is used to evaluate the antidepressant effects of chronic antidepressant treatment in rodent [26]. Appetite in NSF test was affected by CUMS and was improved by XYS and FLU administration. It is well known that the great advantage of herbal medicine is to treat some chronic diseases, thus, to further clarify the effects of XYS treatment on the body weight and behaviors, the time course of the 28–42 d stress model was also performed.

As mentioned in the introduction, the Gln/Glu ratio is purported to reflect the Glu/Gln cycle in neuron-glia communication, which plays a pivotal role in excitatory neurotransmission [33]. Imbalance between Gln and Glu might be associated with MDD through abnormalities of excitatory neurotransmission [34]. Many clinical studies involving patients experiencing depression have demonstrated that the concentrations of these two amino acids fluctuated in plasma and in the brain [34–40]. Proton magnetic spectroscopic evaluation showed increases in the cerebrospinal fluid levels of Glu in depressed patients [41]. Elevated Glu and glycine levels in patients with major depression were also reported [42]. Another study demonstrated that the higher levels of Glu in patients were significantly different from those in healthy volunteers and that the levels decreased as a response to therapy. On the contrary, decreased Gln values based on the results of spectroscopic studies were reported by Auer and colleagues [43]. Interestingly, in agreement with these clinical studies, our current results showed increased Glu and decreased Gln in depressed mice induced by CUMS and these alterations could be effectively restored by the administration of XYS. It has been reported that the levels of glutamine and glutamate (Glu) in the hippocampus in participants at familial risk of depression (FH+) were increased) [44]. In the present study, we also observed an elevated Gln/Glu ratio, which could be explained by impairment in the Glu/Gln cycle. Taken together, these observations suggest that any disturbances in this cycle result in a nonhomeostatic state for Gln and Glu levels and depressive-like behaviors result from such circumstances. Furthermore, the hypothesis of the antidepressant effects of XYS seem reasonable, because imbalance induced by CUMS between Gln and Glu can be normalized by XYS administration.

The actions of glutamate transporters EAAT1–2 have at least two functions, including the clearance of EAA from the synaptic cleft, and the supplying of Glu to glutamine synthetase for Gln synthesis [45]. That is to say, if there were a problem in the EAAT1–2 system, excitotoxicity in the extracellular space and decreased synthesis of Gln would take place. In agreement with this theory, lower rates of EAAT1–2 activity had been considered a cause of depressive disorders [46]. A microarray analysis of specific areas in postmortem cerebral cortex from patients who suffered from MDD showed a significant down-regulation of EAAT1 and EAAT2 [47]. One study showed that the levels of GLAST and GLT-1 could be changed by exposure to stress corticosterone or stress [48]. Another study reported a significant suppression of GLT-1 in the hippocampal and cortical brain regions of helpless animal model [18]. In the present study, our observations of reduced expression of GLT-1 protein and mRNA in CUMS mice were in agreement with those data except GLAST. Our results also indicated a reduction of GLT-1 could be reversed by XYS or FLU treatment. However, several reports showed that chronic mild, predictable stress not only leads to increased glutamate release but also results in EAAT2 elevation [49–51]. Therefore, the directionality of EAAT2 has been somewhat mixed. This likely explains the fact that predictable stress has a beneficial effect on the depressive and anxiety-like behaviors [52, 53]. On the other hand, chronic unpredictable stress decreases EAAT2 levels and which is a similar tendency observed in patients with MDD [18, 47, 54, 55]. To further confirm the results of protein and mRNA expression of two glutamate transporters in CUMS mice, the expressions of GLAST and GLT-1 in the hippocampus were measured by immunohistochemical staining. Interestingly, a similar tendency was also observed and supported by a recent study performed by Chen et al. who reported a decrease in GLT-1 immunostaining in the hippocampus of CUS rats [54]. Previous research reported by Raudensky et al.*,* showed that 10 d CUS (chronic unpredictable stress) elevated GLT-1 immunoreactivity in the dorsal hippocampus, which might be a homeostatic response to regulate or buffer increased extracellular concentrations of Glu [56]. Based on this result, we hypothesized that chronic unpredictable mild stress would lead to a decreased expression of GLT-1 in the CA1, CA3 and DG subregions of the mouse hippocampus, which could be reversed by XYS treatment.

Additionally, in contrast to a human postmortem-investigation [47], we found that 21-d CUMS had no effect on the expression of GLAST, and no change was observed following XYS or FLU treatment. On the other hand, this expression tendency of GLAST in the hippocampus of rat models of stress and depression was also observed [18]*.* Together, these findings indicate that reduced GLT-1 levels might not be a confounding factor caused by the antidepressant medication taken by the patients with MDD, but rather, it can represent a disease-inherent deficit in glutamate uptake. Furthermore, the precise mechanism of action of XYS on the glutamatergic system must be further studied. Particularly, the alteration of functional roles in condition loss of EAATs should be evaluated by using GLT-1 inhibitor or GLT-1^−/−^ mice.

## Conclusion

The present study demonstrates that CUMS causes changes in Glu/Gln cycle, reductions in GLT-1 levels which account for 80% of Glu transport, and produces a depressive-like phenotype. These findings are consistent with a growing number of studies showing markedly abnormal Gln/Glu ratio and glutamate transporter levels in individuals with MDD. Furthermore, we demonstrate that XYS, an herbal prescription, reverses the Glu/Gln cycle ratio imbalance, restores the expression of glutamate transporters and attenuates behavioral consequences of CUMS. Importantly, the present study is the first to demonstrate that changes in the glutamine-glutamate cycle and glutamate transporter GLT-1 expression caused by CUMS can be reversed by XYS. This study sheds new light on targeting pathological changes in the glutamatergic system in depressed subjects using an herbal prescription.

## Abbreviations

AOD: Decreased average optical density
CNS: Central Nervous System
CUMS: Chronic unpredictable mild stress
EAATs: Excitatory amino acid transporters
FLU: Fluoxetine
FST: Forced swim test
GLAST/EAAT1: Excitatory amino acid transporter 1
Gln: Glutamine
GLT-1/EAAT2: Excitatory amino acid transporter 2
Glu: Glutamate
LC-MS/MS: High-performance liquid chromatography-mass spectrometry analysis
MDD: Major Depressive Disorder
NSF: Novelty-suppressed feeding
SPT: Sucrose preference test
TCM: Traditional Chinese Medicine
XYS: Xiao Yao San
